This article has been retracted.

# Discussion on the Transoral Vestibular Approach Endoscopy for TC Patients and the Significance of Serum 25-Hydroxyvitamin D Classification

**DOI:** 10.1155/2022/3425225

**Published:** 2022-04-12

**Authors:** Chunjiang Yang, Leitao Yu, Yong Xiao, Longhong Ouyang, Xiaohua Huang

**Affiliations:** ^1^Department of Head and Neck Surgery, The Second Affiliated Hospital of Nanchang University, Nanchang 330006, China; ^2^Department of Surgery, Yongfeng People's Hospital, Jian 331500, China

## Abstract

In order to discuss the transoral vestibular approach endoscopy through oral vestibular approach in TC and the efficacy of 25(OH)D classification, a total of 110 TC patients from January 2020 to June 2021 are selected. The endoscopic group and the control group are respectively established according to different surgical approaches, with 55 cases in each group. The control group received conventional TC resection, while the endoscopic group received endoscopic assisted TC resection through oral vestibular approach. The differences of intraoperative and postoperative indicators, clinical efficacy, incidence of adverse complications, VAS score, and total satisfaction are observed. TC resection assisted by endoscopy through oral vestibular approach can effectively improve all intraoperative indicators and reduce postoperative pain and has high safety in clinical application. In addition, this study conducted in-depth analysis and classification of serum 25(OH)D index level in postoperative TC patients, indicating that the serum 25(OH)D index level is closely related to prognosis, providing a basis for follow-up clinical monitoring of TC patients' signs and optimization of diagnosis and treatment plans.

## 1. Introduction

Thyroid carcinoma (TC) is a common type of malignant tumor disease in endocrinology and otorhinolaryngology. It mostly occurs in middle-aged people, with many female patients. At present, the incidence is gradually increasing and developing in younger age [1]. The incidence of TC is mainly from the thyroid follicular epithelium. With the progression of the disease, TC in patients' body has different forms, including papillary TC, follicular thyroid carcinoma TC, and medullary TC. At present, the common clinical carcinogenesis is mostly papillary [2]. In clinical practice, surgical resection and lymph node dissection are mostly performed for TC, but the traditional surgical method brings large wounds to the body surface of TC patients. If the follow-up care is improper, scars are easily left after the recovery period, which affects the appearance and brings serious interference to the patients' body and mind [3]. With the improving of the medical profession technical level and popularizing the concept of minimally invasive penetration, it effectively promoted the clinical minimally invasive technology constantly updated, and the oral vestibular into the thyroid gland resection operation for road cavity mirror arises at the historic moment. Compared with the traditional surgery, the trauma of patient airframe is smaller. At present, it has been used to treat hyperthyroidism, benign thyroid tumor, goiter and thyroid nodule benign disease, high clinical efficacy, and satisfaction are achieved, but the efficacy and safety of this operation in TC resection compared with traditional operation are still unclear [4]. In addition, the adjustment of nutritional status after TC resection may have a certain impact on the recovery and prognosis of patients, and THE progression of TC is slower than other malignant tumor diseases, but there is no clear marker to predict and evaluate the prognosis of patients [5, 6]. Based on this, this study conducted a comparative study on the surgical approaches of TC patients and observed their efficacy and conducted a comparative analysis on the prognosis of TC patients based on the nutritional status index 25(OH)D to provide reference data for clinical monitoring of TC patients' signs and effective prognosis evaluation. The results of the study are reported as follows.

A total of 110 TC patients admitted from January 2020 to June 2021 are selected and divided into endoscopic group and control group according to different surgical approaches, with 55 cases in each group. In the endoscopic group, there are 21 males and 34 females, aged from 30 to 66 years, the average is (41.35 ± 5.86) years, with a disease course of 1.2 to 7.0 years, the average is (3.74 ± 1.13) years, with a tumor diameter of 10 to 18 mm, the average is (12.33 ± 1.64) mm, and 24 patients with left-sided disease, and 31 patients with right-sided disease. The mean value of thyroglobulin (Tg) before operation is (137.12 ± 16.91) ng/mL in 34 patients with papillary TC and 21 patients with follicular TC. In the control group, there are 17 males and 38 females, aged from 28 to 65 years, the average is (40.12 ± 5.27) years, and the course of disease is 1–7.5 years, the average is (3.42 ± 1.05) years. The tumor diameter is 11–17 mm, the average is (12.82 ± 1.73) mm. The disease occurred in 21 patients with left side and 34 patients with right side. There are 37 patients with papillary TC and 18 patients with follicular TC, and the mean preoperative Tg is (139.43 ± 17.22) ng/mL. There are no significant statistical differences in gender, age, course of disease, location of disease, TC type, preoperative Tg mean value, and other general data (all *P* > 0.05), which confirmed that the comparison between groups is scientific and reasonable. Inclusion criteria: (1) patients who met TC diagnostic criteria according to preoperative pathological biopsy and imaging detection results and clinical diagnosis [7]; (2) the tumor diameter ranged from 10 mm to 20 mm; (3) all lesions are single; (4) before admission to our hospital, she had not received radiotherapy or chemotherapy. Exclusion criteria: (1) patients with other malignant tumor diseases; (2) complicated with serious organic diseases such as the liver and kidney; (3) drugs affecting vitamin D level and thyroid function are taken within 3 months before admission; (4) patients with surgical contraindications or acute oral inflammation. Serum 25(OH)D index is detected in all patients after operation, and subgroups are established according to different levels of index, which are 25(OH)D insufficient group and 25(OH)D adequate group.

The rest of this paper is organized as follows.  Section 2 summarizes data and methods. In Section 3, the experimental results are given in detail. The analysis of results is presented in Section 4. Conclusion and future work are summarized in Section 5.

## 2. Data and Methods

All patients received general anesthesia before surgery and are placed in supine position after shoulder pads. During surgery, pathological specimens are collected and pathological examination is performed after rapid freezing. The incision is sutured after drainage tube placement. Patients in the endoscopic group received endoscopic thyroid carcinoma resection through oral vestibule, teeth and oral cleaning is performed 1 d before surgery, and general anesthesia is intubated through nasal cavity. After routine preoperative disinfection, dilation fluid (adrenaline and 0.9% sodium chloride solution, ratio: 1 : 200,000) is injected into the anterior part of the neck through oral vestibule. A transverse incision of about 10 mm in length is made for the lower lip of the vestibular cavity of the patient, and the platysma muscle is separated and inserted with a 10 mm puncture needle before the endoscopy is placed. A longitudinal incision of 5 mm is made on both sides of the observation hole, and a 5 mm puncture needle is made after the deep surface of the platysma muscle is separated to complete the puncture, and surgical operations are performed around the puncture hole. Lymph nodes around the affected area are dissected. After surgery, the surgical field of vision is irrigated and hemostatic measures are taken. The incision is sutured without drainage tube. After surgery, oral cavity is cleaned and sterilized with drugs.

The serum level of 25(OH)D is determined by high-performance liquid chromatography-tandem mass spectrometry (HPLC-MS/MS). Index level ≤30 ng/mL is considered as insufficient 25(OH)D, and index level >30 ng/mL is considered as sufficient 25(OH)D [8]. The mass spectrometer (API 320) used in the detection process is purchased from AB SCIEX, Shimadzu series liquid chromatograph is purchased from Shimadzu, Japan, and the detection reagent is purchased from Jinan Yingsheng Biotechnology Co., Ltd. The instrument and test paper are strictly operated according to the corresponding instructions. Observation indicators: changes in intraoperative and postoperative indicators are compared; (2) the clinical efficacy of the two groups is compared; (3) the incidence of adverse complications is compared; (4) visual analogue scale (VAS) scores and total satisfaction are compared after surgery; (5) the 6 months prognosis of patients with different levels of serum 25(OH)D after surgery; (6) spearman analysis of correlation between serum 25(OH)D and prognosis of TC patients.

## 3. Evaluation Criteria

After surgery, the clinical efficacy is evaluated, and significant effect is found: postoperative imaging equipment examination showed no lesion, and Tg value <10 ng/mL; Effective: imaging equipment examination showed that there are some lesions in thyroid tissue, but the diameter of the lesions decreased by ≥30% compared with that before surgery, and the Tg value decreased and changed by more than 25% compared with that before treatment. Ineffective: imaging equipment examination showed that thyroid tissue had lesions and showed no decrease or growth (increase ≥20%) compared with preoperation; Tg value continued to increase or decreased ≤25% compared with pretreatment. Total response rate = (significant effect + effective) cases/total cases × 100%[9].

Postoperative pain is evaluated by VAS scale: 0 is divided into painless, the body can feel the pain but does not affect sleep (1∼3 points), judged to be mild pain; the pain is more obvious and affects sleep, needs to be supplemented by sedative drugs (4∼6) as moderate, and painful, and unbearable, unable to sleep normally (7∼9 points) to determine severe pain, divided into 10 pains [10].

SPSS 26.0 software is used to complete effective processing of the study data [11–14]. The measurement data are tested for normality and homogeneity of variance to satisfy the normal distribution, represented by mean ± standard deviation, independent sample *T* test for intergroup comparison, paired *T* test for intragroup comparison, (*n*, %) for count data, and *x*^2^ test; Kaplan–Meier curve is used to analyze the prognosis of the two groups 6 months after surgery. Spearman correlation coefficient is used to analyze the correlation between serum 25(OH)D and the prognosis of TC patients [15–17].

## 4. The Experimental Results

### 4.1. Comparison of Intraoperative and Postoperative Indicators

The operative time, intraoperative blood loss, and hospital stay in the endoscopic group decreased significantly (all *P* < 0.001), as shown in Table 1.

### 4.2. Compared Clinical Efficacy

The total clinical effective rate of the endoscopic group increased significantly (*P* < 0.05), as shown in Table 2.

### 4.3. Adverse Complications Are Compared

The total number of adverse complications in the endoscopic group is less, but there is no significant statistical difference (*P* > 0.05), as shown in Table 3.

### 4.4. Comparison of VAS Score and Satisfaction

The total clinical satisfaction of endoscopic group increased significantly (*P* < 0.05). VAS score of the endoscopic group decreased significantly (*P* < 0.001), as shown in Table 4.

### 4.5. Prognosis of Patients with Different Levels of Serum 25(OH)D after Surgery Is Compared

Subgroups are established according to the level of serum 25(OH)D after operation, which are 25(OH)D deficient group (*n* = 63) and 25(OH)D adequate group (*n* = 47). The total incidence of adverse events 6 months after surgery in the 25(OH)D sufficient group decreased significantly (*P* < 0.05). The prognosis is shown in Table 1, and the difference curve of adverse events is shown in Figure 1.  Table 5 is 6-month prognosis of patients with different levels of serum 25(OH)D after surgery.

### 4.6. Analysis of the Correlation in TC Patients

Spearman correlation coefficient analysis showed that serum 25(OH)D level is significantly negatively correlated with prognosis in TC patients (*P* < 0.05), as shown in Table 6.

Combined with clinical practice and research, conventional mass resection for TC is usually adopted in the past. Although it is safe, it brings large wounds to the patient's body and increases the risk of postoperative infection to a certain extent. In addition, there are more female TC patients, and large wounds are not conducive to postoperative recovery and healing and may even cause obvious scars. Female patients have more serious troubles. Transvestibular endoscopic thyroidectomy is developed and applied clinically in 2011, which greatly reduced the degree of trauma to patients, effectively improved clinical satisfaction, and is widely used in clinical treatment of thyroid diseases.

The results of this study showed that the operative time, intraoperative blood loss, and length of hospital stay in the endoscopic group are significantly reduced compared with the control group, and the incidence of postoperative adverse complications is effectively controlled. The clinical efficacy is better than that of the control group, which is similar to the results of Feng Ping et al. In addition, this surgical method is minimally invasive and has less trauma to patients, effectively reducing the amount of intraoperative blood loss. This study compared the postoperative pain of patients in the two groups and showed that VAS score in the endoscopic group decreased significantly. The reason may be that the surgical method used in the endoscopic group used ultrasonic knife to remove thyroid malignant tumor, which could effectively stop bleeding after completion of the operation, thus reducing postoperative pain. It is further confirmed that endoscopic thyroidectomy through oral vestibule is superior to traditional thyroidectomy in terms of minimally invasive treatment effect and high safety. In endoscopic thyroidectomy, the recurrent laryngeal nerve is most likely to be damaged when entering the larynx from the recurrent laryngeal nerve, and the injury of the recurrent laryngeal nerve and parathyroid gland should be avoided as much as possible during surgery.

In addition, it has been shown that vitamin D level of patients is closely related to the incidence and progression of malignant tumors, and this index level can reflect the nutritional status of TC patients to a certain extent. Therefore, in this study, serum 25(OH)D level of TC patients after surgery is detected and a subgroup is established around this index. The total incidence of adverse events 6 months after operation in the 25(OH)D sufficient group decreased significantly, and the serum 25(OH)D level is negatively correlated with the prognosis of patients. Related biological and clinical data show that vitamin D can effectively promote cell differentiation and induce tumor cell apoptosis in human body and has an important effect on human immune regulation. The main mechanism of vitamin D transformation into 25(OH)D is the fusion of 25-hydroxylase secreted by human liver. In systemic circulation, 25(OH)D can inhibit tumor cell proliferation and metastasis by binding to vitamin D receptor and controlling the expression of downstream target genes. It is suggested that with the decrease of vitamin D expression level, the weaker the effect of inhibiting tumor cell proliferation and metastasis, the faster the tumor cell proliferation, the greater the possibility of recurrence and metastasis, and the more significant the impact on the prognosis of patients.

## 5. Conclusion

To sum up, the oral vestibular approach joint cavity mirror TC resection applied to clinical practice can effectively shorten the operation time, reduce postoperative pain in patients with trauma to the patient, and reduce the feeling, the clinical curative effect is distinct and conforms to the patients of postoperative cosmetic satisfaction; more patients' postoperative recovery fully confirmed that the operation has high security and worthy of clinical popularization and application. In addition, this study further analyzed the postoperative 25(OH)D level of TC patients and found that low 25(OH)D level is associated with poor prognosis of TC patients, which further confirmed that the application of vitamin D in the prevention and treatment of thyroid cancer has certain clinical guiding significance and provided a basis for the subsequent clinical development of the improvement plan for the prognosis of TC patients.

## Figures and Tables

**Figure 1:** Differences in adverse events 6 months after surgery.

**Table 1:** Comparison of intraoperative and postoperative indicators.

Group	The operation time (min)	Intraoperative blood loss (mL)	Number of dissected lymph nodes (*n*)	The length of time (d)
Group of cavity mirrors (*n* = 55)	75.47 ± 7.32	30.18 ± 4.84	7.03 ± 0.29	5.16 ± 1.05
The control group (*n* = 55)	104.53 ± 10.19	52.62 ± 7.43	6.79 ± 0.26	8.49 ± 2.26
*t*	−17.177	−18.768	1.523	−9.910
*P* value	＜0.001	＜0.001	0.131	＜0.001

**Table 2:** Comparison of clinical efficacy (*n*, %).

Group	Obvious effect	Have the effect	No effect	Total effective rate
Group of cavity mirrors (*n* = 55)	36 (65.45)	13 (23.64)	6 (10.91)	49 (89.10)
The control group (*n* = 55)	21 (38.18)	17 (30.91)	17 (30.91)	38 (69.10)
*x* ^2^	—	—	—	6.652
*P* value	—	—	—	0.010

**Table 3:** Comparison of adverse complications (*n*, %).

Group	Recurrent laryngeal nerve injury	Functional dysfunction of the parathyroid gland	Hypocalcemia	Infection of incision	The total incidence
Group of cavity mirrors (*n* = 55)	2 (3.64)	1 (1.82)	4 (7.27)	1 (1.82)	8 (14.55)
The control group (*n* = 55)	4 (7.27)	2 (3.64)	6 (10.91)	2 (3.64)	14 (25.45)
*x* ^2^	—	—	—	—	2.045
*P* value	—	—	—	—	0.153

**Table 4:** Comparison of VAS score and total satisfaction.

Group	Satisfaction feel quite pleased	Satisfied	Not satisfied	Satisfaction	VAS score
Group of cavity mirrors (*n* = 55)	32 (58.18)	19 (34.55)	3 (5.45)	51 (92.73)	3.34 ± 0.56
The control group (*n* = 55)	18 (32.73)	23 (41.82)	14 (25.45)	41 (74.55)	5.19 ± 0.73
*t/x* ^2^	—	—	—	6.643	−14.912
*P* value	—	—	—	0.010	<0.001

**Table 5:** 6-month prognosis of patients with different levels of serum 25(OH)D after surgery (*n*, %).

Group	Transfer of recurrence	Death	Total incidence of adverse events
25(OH)D deficiency group (*n* = 63)	18 (28.57)	3 (4.76)	21 (33.33)
25(OH)D abundant group (*n* = 47)	6 (12.77)	1 (2.13)	7 (14.89)
*x* ^2^	—	—	4.824
*P* value	—	—	0.028

**Table 6:** Correlation between serum 25(OH)D level and prognosis.

	Adverse prognostic events occurred	
	*r*	*P* value
Serum 25(OH)D	−0.746	0.002

## Data Availability

The simulation experiment data used to support the findings of this study are available from the corresponding author upon request.
